The article "Multimedia Automation Access Control of Big Data Open Resources Based on Blockchain" was published in 2022. Journal: Comput Intell Neurosci.

# Multimedia Automation Access Control of Big Data Open Resources Based on Blockchain

**DOI:** 10.1155/2022/4410075

**Published:** 2022-05-23

**Authors:** Nan Zhao, Hui Su, QingSheng Han, Yan Zhao

**Affiliations:** ^1^Beijing Institute of Economics and Management, Beijing 100102, China; ^2^Unit 78111 of PLA, Chengdu 610011, China

## Abstract

In order to better mine the value of data, the author proposes a research on the automatic access control of big data open resources multimedia based on blockchain and introduces big data access control BBAC-BD (blockchain-based access control mechanism for big data environment). The author designed a strategy management contract based on the Bloom filter, as a probabilistic data structure with extremely high space utilization efficiency and proposed the strategic management contract (PAP CONTRACT) and the strategic decision contract (PDP CONTRACT). In this way, the nontampering, auditability, and verifiability of the access control information are guaranteed; then, the access control method based on smart contracts is adopted to realize the user-driven, whole-process transparent, and dynamic and automatic access control of big data resources. The simulation results show that the greater the ratio of *n*/*k*, the better the optimization effect, and the greater the ratio, the lower the corresponding misjudgment rate, but it will also take up more space costs. At the same time, the true value of the false positive rate is generally less than the theoretical value of the false positive rate. When the performance of Hash (strategy to retrieve) is better, the result of Hash distribution is more uniform. Under the condition of *m* = 3, the misjudgment rate acceptable for the expected use can be achieved, and the increase in the number of Hashes will not bring a significant increase in revenue. Freed from the traditional model of providing access control services based on third parties, solve the problem of transparency of authority judgments; at the same time, through smart contracts, based on the strategy published by the resource owner on the blockchain, realize automatic access control to big data resources; and make the judicial process more flexible and the judgment result more credible. The BBAC-BD mechanism realizes a safe, reliable, and transparent new access control architecture, and it can effectively promote the safe circulation and sharing of big data.

## 1. Introduction

Human society is accompanied by social networks, e-commerce, and mobile communications, and the rise of the Internet of Things, which has entered the era of big data with data volume, big data analysis, and prediction based on distributed computing. This can make decisions more precise of what people are seeing is just the tip of the iceberg of the true value of big data [1]. Smartphones and wearable devices make every change of our behavior, position, and even physiological information become data that can be recorded and analyzed, but these big data are stored and controlled by various government agencies, business alliances, scientific research institutions, and even individuals, and the phenomenon of “data islands” is formed [2]. Interconnect and sharing of these scattered big data, in order to obtain products and services of great value, is an urgent need coexisting in business, scientific research, public services, and other fields [3]. In order to realize big data sharing, it is first necessary to connect separate and decentralized data sources [4]. However, due to the lack of detailed and transparent institutional standards, open policies, and pricing mechanisms between enterprises, scientific research institutions, and government departments, it is difficult to achieve fairness and equality between sharing parties [5]. Data diversification, storage structure, and interaction standards are not uniform, and the lack of a transparent communication environment is also hindering data interaction; the technical architecture of big data access control is shown in Figure 1 [6]. These problems together

r cause data connection difficulties. Therefore, a transparent and open data connection method is urgently needed to record data information, access conditions, standards, and other related information to achieve interconnection. Fundamentally speaking, the issue of “data islands” is mainly related to interest and security issues. The data are kept by a large data platform or other intermediary organization. Once the data are uploaded, the owner loses the right to control the data. Regardless of whether it is a government agency or an Internet company, it is very sensitive to data, and once it is leaked, it will have a great social impact.

The article "Multimedia Automation Access Control of Big Data Open Resources Based on Blockchain" was published in 2022. Journal: Comput Intell Neurosci.

## 2. Literature Review

In response to this research question, the author of [7]aimed at third-party collection and control of personal data security vulnerabilities, leading to the problem of user privacy leakage; a distributed personal data management system based on blockchain is proposed to ensure users own and control their private data. For all blockchain transactions, Ansart et al. are transparently embodied in the public network that leads to the leakage of transaction privacy, and they proposed the use of the Hawk protocol based on smart contracts; the agreement encrypts the communication between the parties to the contract to ensure the absolute security of information [8]. Liu et al. addressed the issue of data security and privacy in the Internet of Things, proposed a lightweight blockchain application suitable for IoT devices, and in the smart home scene, they practiced and verified its security, confidentiality, integrity, and availability [9]. Yin et al. adopted an encrypted smart contract, protected public privacy files through public and private keys, and provided auditing and tracking [10]. In terms of data storage and authenticity verification, Xu, J. et al. made an in-depth discussion on the future impact of the audit industry based on big data analysis and blockchain technology, and studied how to incorporate blockchain into future audit procedures based on the existing theoretical framework [11]. Yu et al. proposed using blockchain to build a secure global named storage system, including the three-tier architecture of the blockchain-based naming system. The naming system is divided into three layers: data layer, routing layer, and blockchain layer [12]. Zhang et al. proposed a method for ensuring the authenticity of microbial sampling robot data based on the bitcoin blockchain, which makes the robot not be interfered by human factors in the process of collecting data, especially the malicious tampering behavior of third-party regulatory agencies [13]. Fan et al. aimed at the three types of credibility problems existing in the current Internet of Things data sharing management and proposed blockchain-based solutions, including a decentralized Internet of Things data sharing architecture and smart contract collection [14]. Ling et al. built an access control architecture for the Internet of Things to provide a more flexible management plan [15]. Bera et al. proposed a resource access control method based on blockchain technology and combined XACML with bitcoin to realize the reliable authority control mechanism based on rules [16]. On the basis of the current research, the author proposes a research on the automatic access control of big data open resources multimedia based on blockchain, using the big data access control BBAC-BD mechanism based on blockchain; it also elaborated and analyzed the basic framework and process of access control in detail. At the same time, for access control strategies based on blockchain transactions and entity attribute information management methods, with the increase of policy rules, the success rate of strategic judgments has decreased, and the BBAC-BD mechanism has realized a safe, reliable, and transparent new access control architecture, and it can effectively promote the safe circulation and sharing of big data.

## 3. Methods

### 3.1. Big Data Access Control Architecture

Big data access control involves the collection, aggregation, management, and control of big data resources. The big data access control architecture is mainly composed of 6 parts: data layer, resource aggregation layer, infrastructure layer, transaction layer, consensus layer, and access control contract layer. Each layer structure cooperates with each other and performs its own duties to form a complete big data access control architecture [17].

1. Data layer: real big data resources, including structured data, unstructured data, and semistructured data distributedly stored in different locations and logically managed by the resource aggregation layer [18];
2. Resource convergence layer: resource management of big data resources based on blockchain technology to realize the convergence of big data resources from different sources. Although real big data resources are in fact distributed and stored by different data owners, but through blockchain technology, it logically forms a unified management of big data resources. The author's research focuses on the access control mechanism, and the resource aggregation layer will not elaborate [19].
3. Infrastructure layer: the blockchain platform provides infrastructure for big data access control. It is the foundation of the whole architecture, and the nodes and minors of the entire network are required to maintain the normal operation of the system. It is the carrier of big data access control platform transactions and smart contracts. The transaction layer, contract layer, and resource aggregation layer are all upper-layer applications based on blockchain.
4. Transaction layer: it includes 4 types of access control transactions: data transaction, strategy transactions, attribute transactions, and contract transactions. Data transactions are used to manage big data resources, which serve at the resource convergence layer. Policy transactions are used to manage access control policies, including the release, update, and sale of strategies to provide data support for PAP CONTRACT at the contract layer. Attribute transactions are used to manage the attributes of entities, including the release, update, and sale of properties to provide data support for the contract layer AA CONTRACT, and contract transactions are used to provide an operating environment for smart contracts, which serve at the contract layer [20];
5. Consensus layer: it mainly includes consensus mechanism, through various consensus algorithms, in order to ensure the consistency and authenticity of access control data among distributed nodes, so as to reach a stable consensus among nodes [21];
6. Access control contract layer: it includes three types of contracts: PAP CONTRACT, PDP CONTRACT, and AA CONTRACT; PAP CONTRACT is used for access control strategy management, PDP CONTRACT is used for access control request judgment, and AA CONTRACT is used for entity attribute management.

The article "Multimedia Automation Access Control of Big Data Open Resources Based on Blockchain" was published in 2022. Journal: Comput Intell Neurosci.

In order to obtain the initial judgment matrix *EQ*=(*eqij*)_*m*×*m*_, there are *m* matrices *E*=(*e*1, *e*2,…, *em*), and the matrix is concentrated in the importance of *ei* and *ej* for binary comparison, which is shown in the following formula:

(1) $$\begin{array}{c} eqij=\left\{\begin{array}{cc} 0, & ei<ej,\\ 0.5, & ei=ej,\\ 1, & ei>ej. \end{array}\right) \end{array}$$

Convert the initial judgment matrix into a fuzzy consistent matrix, which is shown in the following formula:

(2) $$\begin{array}{c} \left\{\begin{array}{c} qij=\frac{qi-qj}{2m}+0.5,\\ qi=\sum_{k}^{m}=1eq_{ik}. \end{array}\right) \end{array}$$

Calculate the weight vector *W*=(*w*_1_, *w*_2_,…,*w*_*m*_)^*T*^ of each evidence of a certain *m* characteristic, which is shown in the following formula:

(3) $$\begin{array}{c} w_{i}=\frac{\sum_{k}^{m}=1qik-0.5}{m\left(m-1\right)/2}. \end{array}$$

Next, the evaluation value matrix of the user behavior characteristic is calculated, and the value on the diagonal of the matrix obtained from the evidence matrix *E*=(*eij*)_*m*×*n*_ and the weight matrix *W*=(*w*_*ij*_)*m* × *n* according to *E* × *W*^*T*^ is the characteristic evaluation value matrix *F*=(*f*1, *f*2,…*fn*). The behavioral credit of the final user is shown in the following formula:

(4) $$\begin{array}{c} \text{current}\_T\left(u\right)=1-F\times W_{f}^{T}=1-\sum_{i=1}^{n}fiwi. \end{array}$$

current_*T*(*u*) represents the user's current credit rating, and *W*_*f*_=(*W*_*f*1_, *W*_*f*2_,…, *W*_*fn*_) represents the weight of the user's behavioral characteristics. When the user logs in for the first time to perform access control, the system will generate the first historical credit according to the user's software and hardware operations: History_*T*_1_(*u*)=Current_*T*_1_(*u*). As the number of visits increases gradually, the user's historical credit needs to be gradually changed according to the passage of time as shown in the following formula:

(5) $$\begin{array}{c} \text{History}\_T\left(u\right)=\left\{\begin{array}{c} 0,\;n=0,\\ \sum_{i=1}^{n}\left(Final\_Ti\left(u\right)\times ti\right),\;n>0,\\ \sum_{i=1}^{n}ti. \end{array}\right) \end{array}$$

Final_*T*_*i*_(*u*) corresponds to the user's final credit at the end of each visit and *t*_*i*_ records the access time. This parameter calculates the total time from the user's login to the end of the user's exit from the system. When *n* = 0, it means that the user has logged into the system for the first time and has no corresponding historical credit value. When a user visits for the first time, there is no historical credit, and the recommended credit will have a certain reference value. The user's recommended credit is calculated based on the credit between the user and other service organizations. Assuming that there are *n* credible access organizations *s*=(*s*_1_, *s*_2_,…, *s*_*n*_), *T* and *N* representing the historical credit value and the number of successful visits of users of service organizations *s*_*i*_ and *u*_*i*_, respectively, then the expression of the recommended credit is shown in the following formula:

(6) $$\begin{array}{c} \text{Recommend}\_T\left(u\right)=\left\{\begin{array}{cc} 0, & n=0,\\ \frac{\sum_{j=1}^{n}\left(Nj\times T_{ui}^{si}\right)}{\sum_{j=1}^{n}Nj}, & n>0. \end{array}\right) \end{array}$$

There is a competitive relationship between the chain generated by the honest node and the chain generated by the attacker. When the honest node is ahead, the chain of the honest node is extended by one block; otherwise, the chain of the attacker is extended by one block. The attacker successfully fills the gap behind *z* blocks, which is similar to the gambler bankruptcy problem, and then the attacker fills the gap and catches up with the honest chain. The probability is shown in the following formula:

(7) $$\begin{array}{c} q_{z}=\left\{\begin{array}{cc} 1, & p\leq q,\\ {\left(\frac{q}{p}\right)}^{z}, & p>q, \end{array}\right) \end{array}$$

where *p* represents the probability of an honest node gaining ownership of the next node, *q* represents the probability of an attacker gaining ownership of the next node, and *qz* represents the attacker filling the gap *z* blocks behind. When *p* > *q*, the probability of the attacker successfully attacking the next block decreases with the increase of *z*. Assuming that honest blocks take the average expected time to generate a block, the potential progress of the attacker is calculated according to the Poisson distribution, and the expected value is shown in the following formula:

(8) $$\begin{array}{c} \lambda =z\frac{q}{p}. \end{array}$$

In order to calculate the probability that the attacker will generate nodes and catch up with the honest nodes in the chain when the attacker is behind, the probability is *pz*. We compare the Poisson distribution of blocks obtained by the attacker with the potential attack speed and the probability that the attacker can catch up with the honest nodes. The probabilities are multiplied to obtain the following formula:

(9) $$\begin{array}{c} p_{z}=\sum_{k=0}^{\infty }\frac{\lambda^{k}e-\lambda }{k}\cdot \left\{\begin{array}{cc} {\left(\frac{q}{p}\right)}^{\left(z-k\right)}, & k\leq z,\\ 1, & k>z. \end{array}\right) \end{array}$$

After simplification, the formula is

(10) $$\begin{array}{c} p_{z}=1-\sum_{k=0}^{z}\frac{\lambda k_{e}-\lambda }{k}\cdot \left(1-{\left(\frac{q}{p}\right)}^{\left(z-k\right)}\right)=1-\sum_{k=0}^{z}\frac{{\left(zq/p\right)}^{k}e-zq/p}{k}\cdot \left(1-{\left(\frac{q}{p}\right)}^{\left(z-k\right)}\right). \end{array}$$

The article "Multimedia Automation Access Control of Big Data Open Resources Based on Blockchain" was published in 2022. Journal: Comput Intell Neurosci.

### 3.2. BBAC-BD Workflow

In the BBAC-BD (blockchain-based access control mechanism for big data environment) proposed by the author, the access control workflow is an extension of the standard ABAC model workflow. The access control workflow can be divided into two phases: the preparation phase and the execution phase. The preparation phase is mainly for the management of access control strategies and attributes, including the release, update, and withdrawal of policies and attributes and the response to the results of the policy and attribute query, and the execution phase is mainly for the judgment, response, and execution of the access request [22].

1. Preparation stage: from the property release direction to the blockchain, release property, and property relationship information, AA (attribute authority) CONTRACT collects and integrates attribute information in blockchain transactions in advance, for PEP (policy enforcement point) CLIENT and PAP (point administration point) CONTRACT, from the policy release direction, the access control policy is released in the blockchain. PAP CONTRACT combines attribute information to describe, collect, and integrate access control strategies in blockchain transactions, for PDP (policy decision point) CONTRACT to make an access request decision.
2. Execution stage: when PEPCLIENT receives a request from a user to perform a certain operation on a certain resource, PEPCLIENT analyzes the subject, object, and operational semantics of the original access request, generates an attribute-based access request AAR based on the attribute information obtained from AACONTRACT, sends AAR to PDP CONTRACT, PDP CONTRACT queries PAP CONTRACT for the access control policy set related to the requested big data resource, makes an access control decision, and sends the judgment result response back to PEP CLIENT. According to the response result by PEP CLIENT, authorize access to big data resources, since the access control policy is stored in the blockchain, policy information is verifiable, traceable, and nontamperable to anyone. The access control of big data resources gets rid of the traditional centralized access control management, possible single points of failure, and transparency of access control decisions. It realizes the distributed management of the access control strategy and effectively improves the robustness and credibility of the system. In addition, the decision process of the access control strategy is realized through the form of smart contract, with no need for the involvement of a third-party central agency, and avoids the possible ultravires behavior of the third-party center, based on the blockchain system to realize the automatic judgment of access control under consensus. It is a truly decentralized access control mechanism, which meets the access control management requirements of big data resources [23].

The article "Multimedia Automation Access Control of Big Data Open Resources Based on Blockchain" was published in 2022. Journal: Comput Intell Neurosci.

### 3.3. Transaction Storage in the Blockchain

In the blockchain, data are stored in the blockchain in the form of transactions, we use the form of transactions in the blockchain to manage access control policies, the transaction data in the block are stored in the data structure of the Merkle tree based on the HashHash algorithm, and the transaction data of inconsistent size are mapped into a fixed-size character string through a HashHash algorithm, stored on the leaf nodes of the Merkle tree. The nonleaf nodes of the Merkle tree store the HashHash values of its child nodes. The blockchain includes physical accounts, data blocks, transaction set data, and configuration data. The data view relationship between them is shown in Figure 2.

1. Physical account: it is the initiator of various transaction requests and the owner of related data in the blockchain. It is the actual owner of the data resources in the access control mechanism and has a pair of public and private keys generated by the PKI system. In the system, the account is uniquely identified by the public key, and the transaction data published by the resource owner need to be signed by the entity account with a private key for other users to verify the authenticity of transactions in the block [24];
2. Data block: it is the underlying data in the blockchain network, and multiple blocks together form a chain structure, persist the transaction processing results within a certain period of time in an immutable form.
3. Transaction set data: it is based on the access control mechanism of the blockchain and stores data for performing actual business activities, including access control transactions and smart contract transactions. Access control transactions are used for the management of access control policies; it mainly covers the release, update, and cancellation of policy information in policy management. Smart contract transactions are used in the decision process of access control, in response to access requests and generating access control responses. Issuing transactions on the blockchain requires tokens that consume a certain amount of data, as the user's expenses for using blockchain services.
4. Configuration data: it is the configuration information required for the normal operation of the blockchain system, including configuration information such as protocol version number and communication node information.

The article "Multimedia Automation Access Control of Big Data Open Resources Based on Blockchain" was published in 2022. Journal: Comput Intell Neurosci.

### 3.4. Smart Contract for BBAC-BD

(1) Strategic management contract (PAP CONTRACT).

The flow of the PAP CONTRACT is shown in Algorithm 1.

PAP CONTRACT algorithm flow description.

Analyze the AAR to obtain the requested resource attribute information rttrTuple; traverse the strategic transaction data blocks in each block of the blockchain; obtain the attribute Bloom filter (BF) corresponding to the strategy transaction data block. According to the Hash function corresponding to the BF, calculate the Hash value corresponding to rttrTuple. If the Hash value obtained by calculating rAttrTuple and the corresponding bit in BF are all 1, then add the strategy in the data block in RELEVANT_POLICY_SET; otherwise, there is no rttrTuple related strategy in the data block. When the traversal of strategy transactions in all blocks is completed, return resource-related policy set RELEVANT_POLICY_SET to PDP for permission judgment.

(2) The strategy decision process is carried out by the strategy decision contract (PDP CONTRACT), and the contract flow is shown in Algorithm 2.

PDP CONTRACT algorithm flow description.

Put all pending decisions into UNKNOWN_SET, as a predecision strategy set; traverse the predecision strategy; and get 4 strategy decision result sets:

PERMINT_RESULT_SET DENY_RESULT_SET UNSATISFY_RESULT_SET UNKNOWN_RESULT_SET. According to the judgment result set, the final judgment result of the AAR request is obtained: if there is a conflicting judgment result, the final judgment result is obtained after the conflict is processed, and conflict handling can be based on the principle of affirmative priority or negative priority for conflict resolution.

## 4. Results and Analysis

### 4.1. Strategy Retrieval Efficiency Test

This experiment is aimed at the management method based on the Bloom filter strategy and performed testing on the optimization effect of strategy retrieval efficiency. In the experiment, matching query tests were performed on test sets of different query scales, set different parameters for the Bloom filter to test the error rate and retrieval delay, which were used to evaluate the impact of different parameters of the Bloom filter on retrieval performance. The calculation method of single time delay is total time delay/total number of matches. The optimization effect is mainly through the strategic management contract. The retrieval delay of the strategy is measured. The smaller the delay, the higher the execution efficiency, and the better the search optimization effect. From the test results of Tables 1 and 2, we can see that the larger the ratio of *n*/*k*, the better the optimization effect, and the larger the ratio, the lower the corresponding misjudgment rate, but at the same time, it will take up more space and cost. At the same time, the true value of the false positive rate is generally less than the theoretical value of the false positive rate [25].

The article "Multimedia Automation Access Control of Big Data Open Resources Based on Blockchain" was published in 2022. Journal: Comput Intell Neurosci.

The results of Figures 3 and 4 show that, when the performance of Hash is better, that is, the result of Hash distribution is more uniform, under the condition of *m* = 3. The misjudgment rate acceptable for the expected use can be achieved, the increase in the number of Hashes will not bring a significant increase in revenue. Therefore, when conditions permit, try to expand the value of n/*k* and can effectively improve query performance. This is mainly due to the Bloom filter's attribute keyword filtering process of policy detection, the retrieval time is less affected by the scale of the strategy set, so compared to the traversal retrieval process, strategy retrieval and matching based on the Bloom filter can achieve high performance and strategy retrieval based on the Bloom filter can effectively save cache space, reduce the number of requests to the cache, and improve the efficiency of strategy query and the isolation of strategy management services.

### 4.2. Strategy Decision Function Test

In order to verify the effectiveness of the BBAC-BD access control mechanism, the author under different scales of strategies, judgment function of access control strategy based on smart contract, performed a functional test; the test content includes the efficiency of the strategy decision and the success rate of the decision result. The PolicySamples of 1 to 5 groups correspond to 1000, 2000, 3000, 4000, and 5000 single strategy test set samples, respectively. The test set sample constructs 800 different access requests for 80 user identities; each logo has an average of 5 attribute values, and each request is sent randomly 5 times. The strategy decision delay is obtained by calculating the average response delay of all requests as shown in Figures 5 and 6.

As can be seen from Figure 5, the strategy decision delay is directly related to the strategy scale, with the increase of strategy rules, the delay of access control decision has increased significantly. At the same time, it can be seen from Figure 6 that, as the strategy rules increase, the strategy decision success rate decreases.

The article "Multimedia Automation Access Control of Big Data Open Resources Based on Blockchain" was published in 2022. Journal: Comput Intell Neurosci.

## 5. Conclusion

The author proposes a research study on the automatic access control of big data open resources multimedia based on blockchain. The author uses the big data access control BBAC-BD mechanism based on blockchain. It also elaborated and analyzed the basic framework and process of access control in detail. At the same time, access control strategies based on blockchain transactions and entity attribute information management methods explain that, with the increase of strategy rules, the success rate of strategy decisions decreases. The BBAC-BD mechanism implements a safe, reliable, and transparent new access control architecture, which can effectively promote the safe circulation and sharing of big data. Through smart contracts, based on the strategy released by the resource owner to the blockchain, the automatic access control of big data resources is realized, the judgment process is more flexible, and the judgment results are more credible. The BBAC-BD mechanism is safe, reliable, and transparent. The new access control architecture can effectively promote the safe circulation and sharing of big data. This is because there are some conflicting strategies in the strategy set. For conflicting strategies, the strategic judgment contract cannot get a consistent judgment result, it should be noted that the author has not yet introduced the strategy conflict handling part into the strategy judgment contract, the conflict resolution has not been effectively resolved, and this part of the content will continue to be improved in the follow-up research work.

## Figures and Tables

**Figure 1:** Data access control technology architecture.

**Figure 2:** The relationship between data view entities in the block.

**Figure 3:** Comparison of strategy retrieval performance.

**Figure 4:** M value affects the accuracy of retrieval results.

**Figure 5:** Comparison of strategy decision performance.

**Figure 6:** Comparison of the success rate of strategy decision results.

**Algorithm 1:** Strategy management contract (PAP CONTRACT).

**Algorithm 2:** PDP CONTRACT.

**Table 1:** Strategy retrieval test results 1.

Serial number	*n*/*k*	*m* test value	*M* optimal value	Query size	True false positive rate	Theoretical misjudgment rate	Total delay	Single time delay
1	20	3	14	4000	0.1975	0.2721	432	0.118
2	20	3	14	8000	0.1869	0.2721	798	0.079
3	20	6	14	4000	0.0321	0.0331	762	0.198
4	20	6	14	8000	0.0298	0.0331	1484	0.187
5	20	14	14	4000	0.0074	0.0076	985	0.257
6	20	14	14	8000	0.0095	0.0076	2062	0.255
7	20	20	14	4000	0.0029	0.0141	1247	0.332

**Table 2:** Strategy retrieval test results 2.

Serial number	*n*/*k*	*m* test value	*M* optimal value	Query size	True false positive rate	Theoretical misjudgment rate	Total delay	Single time delay
8	20	20	14	8000	0.0098	0.0141	2 462	0.328
9	10	3	7	4000	0.9356	1.7451	484	0.124
10	10	7	7	4000	0.792	0.891	I 134	0.285
11	5	3	3	4000	9.12	9.21	837	0.229
12	2	1	1	4000	39.51	39.29	762	0.192
13	2	2	1	4000	39.76	40.12	812	0.203

The article "Multimedia Automation Access Control of Big Data Open Resources Based on Blockchain" was published in 2022. Journal: Comput Intell Neurosci.

## Data Availability

The data used to support the findings of this study are available from the corresponding author upon request.
